RETRACTED

# Analysis on frosting of heat exchanger and numerical simulation of heat transfer characteristics using BP neural network learning algorithm

**DOI:** 10.1371/journal.pone.0256836

**Published:** 2021-09-02

**Authors:** Bo Yu, Yuye Luo, Wenxiao Chu

**Affiliations:** 1 State Key Laboratory of Air-conditioning Equipment and System Energy Conservation, Zhuhai, Guangdong, China; 2 Key Laboratory of Thermal-Fluid Science and Engineering, Ministry of Education, Xi’an Jiaotong University, Xi’an, Shaanxi, China; Ministry of Natural Resources North Sea Bureau, CHINA

## Abstract

The study is aimed at the frosting problem of the air source heat pump in the low temperature and high humidity environment, which reduces the service life of the system. First, the frosting characteristics at the evaporator side of the air source heat pump system are analyzed. Then, a new defrost technology is proposed, and dimensional theory and neural network are combined to predict the transfer performance of the new system. Finally, an adaptive network control algorithm is proposed to predict the frosting amount. This algorithm optimizes the traditional neural network algorithm control process, and it is more flexible, objective, and reliable in the selection of the hidden layer, the acquisition of the optimal function, and the selection of the corresponding learning rate. Through model performance, regression analysis, and heat transfer characteristics simulation, the effectiveness of this method is further confirmed. It is found that, the new air source heat pump defrost system can provide auxiliary heat, effectively regulating the temperature and humidity. The mean square error is 0.019827, and the heat pump can operate efficiently under frosting conditions. The defrost system is easy to operate, and facilitates manufactures designing for different regions under different conditions. This research provides reference for energy conservation, emission reduction, and sustainable economic development.

## Introduction

Energy and environmental issues brought about by increasing energy consumption have attracted increasing attention. According to statistics, in China, the building energy consumption has reached 28%-30% of the total energy consumption, of which, 56%-58% is the energy consumption of air-conditioning and heating [1]. The demand for environmentally friendly clean energy and high-efficiency energy technologies has increased globally, due to the shortage energy resources [2]. A heat pump is a device that can obtain low-grade energy from the air, water, or soil, and convert it to high-grade heat energy through electric power [3]. It has attracted much attention due to their "high efficiency" and "relatively low cost". Among them, air source heat pumps are popular in the market because of their convenience and low installation costs [4]. However, in many regions, especially in the high-humidity southern China, the heating effects are not ideal under extreme climate conditions, and other auxiliary measures are often needed to achieve the desired effects [5]. Therefore, to develop air source heat pump devices with good heating effects under extreme climatic conditions is necessary.

RETRACTED

Air source heat pump is a device that uses air as a low-grade heat source to obtain hot water or hot air from it [6]. It not only has high energy efficiency, but also reduces heating energy consumption and environmental pollution. However, severe frosting occurs on the evaporator side resulting from the strong cold air in the north [7], which not only increases the heat transfer resistance of the evaporator, but also increases the wind resistance of the heat exchanger. As a result, the evaporation temperature and condensation temperature decrease, and heating capacity and the energy efficiency ratio decline [8], severely restricting the promotion of air source heat pumps in different regions [9]. Air source heat pump is a device that uses air as a low-grade heat source to obtain high-grade heat, it is important heating equipment. Compared with gas heating or electric heating, it not only has a high primary energy ratio, but also reduces energy consumption and environmental pollution. Therefore, it is widely used in the middle and lower reaches of the Yangtze River and the surrounding areas. Changsha is a typical representative, where the average temperature is low and the relative humidity is high in winter. Therefore, to solve the frosting problem at a low temperature has become urgent.

The innovations of this research are: (I) The concept of ideal minimum defrosting energy is proposed, as well as the calculation method of the minimum auxiliary heat for defrosting; (II) Aimed at defrosting, a front-mounted defrosting heat pump system and a leap-type anti-defrosting heat pump system are proposed. (III) the thermodynamics and heat transfer performance of front-mounted defrost heat pump are simulated. The main contributions of this study are as follows. First, defrost is realized without affecting the heat capacity of the heat pump. Under one atmospheric pressure, the defrosting requires surface temperature higher than 0 degrees under any conditions. In this study, the evaporating side of the heat pump is equipped with an electric auxiliary heating device to include the auxiliary heat into the thermal cycle, which increases the evaporating temperature. As a result, the condensation side generates more heat. Secondly, aimed at the easy frosting under low temperature and high humidity, especially the reduced heat capacity during defrosting, the frosting characteristics at the evaporator side are summarized. Then, a new defrosting system is proposed, and its thermodynamics and heat transfer performance are simulated.

RETRACTED

### Related work

The frost layer can be regarded as a porous medium, composed of ice crystals and air. Related scholars have observed the growth of frost from a microscopic point of view, using the microscopic photography. It is found that, the frosting process is divided into three stages: frost crystal growth period, frost layer growth period, and frost layer mature period [10]. The current research on the characteristics of the frost layer mainly focuses on the density, structure, the thermal conductivity, and the relationship between them. Pan et al. (2017) believed that, when the density of the frost layer increases, the thermal conductivity also increases [11]. Work and Lian (2018) developed a frost layer model based on the frost pillar model, and proposed the equation expressing the relationship between the predicted frost layer thickness and its adhesion speed, as well as the equation expression the relationship between the frost layer density and the effective thermal conductivity [12]. Song and Dang (2018) proposed a complex model to analyze the dynamic distribution characteristics of the thermal conductivity, density, and temperature during the frost layer growth process. He pointed out that, the thermal conductivity of the frost layer is not just a pure density function, and it also includes many other factors [13]. Zhang et al. (2021) made certain amendments to the water vapor penetration process and boundary conditions in the porous medium in the frost layer. They studied the influence of air humidity, temperature, and air velocity on the formation of the frost layer, and the density distribution inside of the frost layer [14]. In addition, Mahvi et al. (2021) believed that, there are many models to predict the characteristics of the frost layer. Thanks to the large differences between the models, to adopt which model is determined by evaporator structure, material, surface condition, wall temperature, air flow rate, humidity and other specific conditions [15].

To analyze the defrosting characteristics of the evaporator, it is necessary to accurately judge the initial condition of defrosting, that is, the frosting status on the surface of the evaporator [16]. Many scholars have conducted experimental research on simple geometric shapes, such as flat plates, cylinders, and other structures. Spötl et al. (2021) explored the influence of working conditions on the growth of frost layer. Aimed at the frosting on a horizontal cylindrical surface, they found that, when the humid air temperature changes between 9.9°C to 20.3°C, the frost layer thickens with the temperature [17]. Additionally, Jansons et al. (2021) reached a consistent conclusion that, the thickness of the frost layer and the quality of frost increase with the humidity of the air, but decrease with the increase of the wall temperature [18]. Lei et al. (2021) investigated the frosting process on the aluminum surface under laminar flow conditions. They observed that, near the air inlet end, the frost layer thickness and frost quality are larger than the air outlet end [19]. Hosseini et al. (2021) summarized the empirical equations of frost layer thickness, frost layer density, and thermal conductivity through experiments [20]. Zhou et al. (2021) established a steady-state distributed parameter model with an air source heat pump unit as the research subject, and established a dynamic distributed parameter model by regarding the frosting process as a quasi-dynamic process. The calculated results were compared with the experimental data, and the influence of temperature and humidity on the amount of frost and system performance was analyzed [21].

RETRACTED

The current defrosting methods mainly include reverse cycle defrosting method, hot gas bypass defrosting method, and electric auxiliary thermal defrosting [22]. Qu et al. (2017) studied the suction and discharge pressures of the compressor during the reverse cycle defrosting. They found that, during the reverse cycle defrosting process, the sudden reversal of the four-way reversing valve will not only affect the suction and discharge pressures, but also cause mechanical loss of the compressor [23]. Li et al. (2018) studied the hot gas defrosting process of an air source heat pump, and understood the dynamic changes of the power consumption of the heat pump, the refrigerant flow parameters, the suction and discharge parameters of the compressor, and the wall temperature [24]. Song et al. (2020) established the equation of water evaporation based on Lews number, and analyzed the energy consumption of heat pump defrosting. The defrost energy consumption was measured through experiments, and it was found that, only 20% of the energy consumption was used for defrosting, and the remaining 80% of the energy was transferred to the heat exchanger and surrounding air through dissipation [25]. Above, related scholars have done a lot of research on the mechanism and characteristics of frosting, with much reliable experimental data obtained. Many empirical equations have been put forward about the growth characteristics and physical properties of the frost layer, and various mathematical models have been established to predict the growth of frost layer. However, there are still few studies on heat pump defrosting, and there are many issues that need to be further studied.

RETRACTED

In the past 50 years, a lot of and fruitful research has been conducted on the frosting mechanism and frosting characteristics of heating devices, with various mathematical models established to predict frost layer growth and heat exchanger performance. However, despite the progress in the mathematical models on defrosting process of air source heat pumps, there are few studies on the defrosting of heat pumps. It is a basic fact that frost will form when the air temperature is lower than 0 degrees. The traditional defrosting methods are all at the expense of reducing the heat capacity of the heat pump, and no longer meet users’ heating needs. As a result, people will look for and purchase other electric heating devices, resulting in more consumption of high-grade energy. In view of the easy frosting problem of the air source heat pump system in the low temperature and high humidity environment, in this study, the frosting characteristics at the evaporator side are analyzed. Then, a new defrost system is proposed, and its thermodynamics and heat transfer performance at the evaporator side are simulated.

## Research methodology

### Neural network control system

Dimensional analysis is a physical research method based on dimensional theory. It only needs to understand the basic laws of the physical process, and does not require to delve into the details of its internal process. Essentially, it describes the consistency of the dimensions in the differential equations. Dimensionless quantity generally refers to the ratio of several similar physical quantities or the dimensionless similarity criterion of different physical quantities. Based on the dimensional theory, the error of predicting the amount of frosting is 18.4% [26]. In the study, the original dimensionless correlation equation of frosting amount is improved by combining dimensionless parameters with neural network. At the same time, the traditional neural network algorithm is optimized, so that the improved model can be used to predict the amount of frosting under multi-working conditions. Moreover, it has a smaller error compared with the original dimensionless correlation equation (with an error of 18.4%). The Birkingham method is adopted [27], and four physical dimensions of time, length, mass, and temperature in the international unit are taken as the basic dimensions. Then, the following dimensionless criteria are derived.


$$X_{1}=t_{a}/t_{s},X_{3}=L/D_{e},X_{3}=\omega \tau /D_{e}$$ (1)

$$X_{4}=ma,X_{5}=mf_{rv}3/(\sigma d_{eq}^{2})$$ (2)

Where *m*_*fr*_ is the amount of frosting of the heat exchanger along the horizontal unit tube length; *t*_*α*_ is the air dry bulb temperature of the heat exchanger coil; *t*_*s*_ is the outer surface temperature of the heat exchanger tube wall; *w* is the front wind speed of the heat exchanger coil along the airflow direction; *L* is the length of the fin along the airflow direction; *σ* is the heat flux density on the *τ* inner surface of the heat exchange tube; *m*_*α*_ is the air moisture content of the sweeping heat exchanger coil; *τ* is the running time (hours); *D*_*e*_ is the equivalent diameter of the air circulation section. Based on above parameters, the neural network structure is used, and the amount of frost is expressed as follows.


$$m_{f}=\frac{\theta D_{e}^{2}}{w^{3}}(\overset{\sigma }{\underset{j=1}{\sum }}w_{1,j}h_{j}+b_{2})$$ (3)

This method may complicate the network, thereby increasing the training time of the network and prone to overfitting [28]. To obtain a more accurate BP network, a three-layer BP neural network is selected when designing the BP network. As shown in Fig 1, they are the input layer, the hidden layer, and the output layer. The input layer has 4 neurons, and each neuron is multiplied by the corresponding weight, and the results is then passed to the next layer through the transfer function. Similarly, the hidden layer is multiplied by the corresponding weight, and the result is passed to the output layer through the transfer function [29]. The mathematical expressions of the hidden layer and the output layer of the three-layer neural network is are as follows.

RETRACTED

**Fig 1:** Dimensionless parameters-BP neural network model structure.


$$h_{j}=g(\sum_{p=1}^{p}u_{jp}x_{p}+b_{1,j}),j=1,2,\ldots J$$ (4)

$$y_{j}=g(\sum_{j=1}^{J}w_{ij}h_{j}+b_{2,j}),j=1,2,\ldots I$$ (5)

Where *b*_*1*,*j*_ and *b*_*1*,*j*_ are the biases of the hidden layer and the output layer, respectively; *b*_*1*,*j*_ and *w*_*ij*_ are the weights between the input layer and the hidden layer, and between the hidden layer and the output layer, respectively. Three common transfer functions g(x) are used then, defined as follows.


$$g_{line}(x)=x$$ (6)

$$g_{\log}(x)=1/1+e^{-x}$$ (7)

$$g_{\tan}(x)=2/(1+e^{-2x})-1$$ (8)

Finally, the non-dimensional parameter-neural network model, used to predict the frosting amount, can be abbreviated as follows.


$$\pi_{5}=f(\pi_{1},\pi_{2},\pi_{3},\pi_{4})$$ (9)

Neural network parameter settings: (I) Network nodes: the number of nodes in the input layer of the network is the number of characteristic factors (independent variables) of the system, and the number of nodes in the output layer is the number of system targets. The number of hidden nodes is generally set as the 75% of the number of nodes in the input layer. If the input layer has 7 nodes and the output layer has 1 node, the number of nodes in the hidden layer can be set to 5, and then a 7-5-1 BP neural network model is established. (II) Initial weight: in the program, a random generator program is set to generate a set of random numbers ranging from 0.5 to +0.5 as the initial weight of the network. (III) Minimum training rate: the training rate is determined by experience. A greater training rate means there are greater changes in the weight, and the convergence is faster. However, if the training rate is too large, it will cause the system to oscillate. Therefore, the value is generally 0.9. (IV) Dynamic parameters: empirically, the dynamic coefficient is generally between 0.6 ~ 0.8. (V) Allowable error: generally, when it is between 0.001~0.00001, the iterative calculation is terminated. (VI) Other parameters: Sigmoid is used to adjust the form of neuron excitation function, generally between 0.9 and 1.0. The number of iterations is generally 1000. Since the neural network cannot guarantee the convergence of the iteration results, when the iteration results do not converge, the maximum number of iterations is allowed.

### Model algorithm optimization

To obtain a reliable and effective network for the trained non-dimensional parameter-neural network correlation, as shown in Fig 2, the control steps are as follows. (1) The temperature and humidity of the environment are recorded, together with the structure parameters and freezing medium of the heat exchanger. With dimensionless parameters X1~X4 as input, a neural network sample training database is established to predict the amount of frost; (2) The preprocessing of neural network, including normalization, initial value setting, determination of the number of neurons in the hidden layer, and error calculation; (3) To train the neural network. Adaptive frosting process control algorithm, with the best hidden layer and the best algorithm selected to automatically adjust the learning rate. (4) To test whether the established neural network is reliable. With the given environmental variables, and heat exchanger structure parameters as input, the amount of frosting is calculated, which is then compared with the known test value; (5) In reference to the previous four steps and the designed heat pump defrost control system, an adaptive defrost heat pump system is established, based on the analysis of heat transfer energy of the frost layer and the ideal minimum defrosting energy theory.

RETRACTED

**Fig 2:** Flow chart of adaptive network control algorithm to predict the amount of frost.

The adaptive network control algorithm takes into account the climate characteristics, the types of freezing media, and the structural size of the heat exchanger, providing a basis for the control of the auxiliary heat during the defrost process [30]. The specific steps of the control algorithm are as follows. Step1: 6 kinds of refrigerants (R12, R134a, R22, R410A, R407C and R600a) are used, and the frosting amount under different heat exchanges and in different regions is recorded, as well as the temperature and humidity of the local environment and the structural parameters of the heat exchanger. Then, the sample database is established with dimensionless parameters X1~X4 as the input and the dimensionless parameter X5 of the frosting amount as the output, to predict the frosting amount; step2: the preprocessing of the neural network. The samples of the database are trained, including normalization, initial value setting, determination of the number of nodes in the hidden layer, and error calculation. If the error satisfies the set value, proceed to the next step, otherwise, return to the initial value setting; step3: training of the neural network. the optimal hidden layer and the optimal algorithm are used to automatically adjust the learning rate. Then, the neural network used to predict the amount of frost is basically established; step4: it is tested whether the neural network of the amount of frost is reliable. With environmental variables, heat exchanger structure parameters, etc. as the input, the amount of frost is calculated and compared with the known test value. If the error is within the given range, it proves that the trained neural network is reliable. If the error is too large, it requires to return to the third step to continue to select different algorithms and learning rates; step5: above, an adaptive defrost heat pump system is ultimately established. The control steps can be summarized as adjusting the amount of supplemental heat to enable the heat pump to run efficiently in winter. The fifth step is based on the first four steps to adaptively predict the amount of frost.

Previous scholars mostly use the following empirical equation to determine the number of hidden layers.


$$i=\sqrt{p+k}+m$$ (10)

Where *i*, *p*, *and k* are the number of hidden layers, input layers, and output layers, and *m* is a constant from 0 to 1 selected based on experience.

### Mathematical model of heat exchanger

Fig 3 is a flow chart of the mathematical simulation model of the air source heat pump unit with an defrost device, including three parts, namely, the environmental working condition model, the heat pump main component model, and the defrost device model. Among them, the environmental working condition module establishes mathematical models for different working conditions. The heat pump is mainly composed of the evaporator, the condenser, the capillary tube, and compressor. The defrost module mainly calculates the required minimum defrost auxiliary heat, based on the amount of frost and the ideal minimum anti-defrost energy. It enables future researchers to choose modules according to their own conditions [31].

RETRACTED

**Fig 3:** A simulation model of defrost heat pump system.

Fig 4 is a flow chart of a modularized computer simulation model. Users can analyze and predict the steady-state and dynamic performance of the heat pump according to the flow chart. In the calculation, provided that, the frosting process is a quasi-static process. To calculate the dynamic changes of the heat pump system, the evaporating temperature changing with time is used as the dynamic time variable, to participate in the cyclic calculation until the output is obtained.

**Fig 4:** A flow chart of a computer simulation model of the defrost heat pump system.

The freezing medium is uniformly sent to each branch fin heat exchange tube through the throttling and evaporation of the capillary tube, to absorb the heat of the air from the sweeping fin tube. Then, it becomes refrigerant vapor and returns to the compressor to participate in a second cycle. The cooled can be sent to the air-conditioned room after being treated to reach the appropriate temperature and humidity. When the heat transfer coefficients of the fluids on both sides of the heat exchanger differ greatly, that is, the freezing medium and the air, it is needed to add fins to the fluid with a smaller heat transfer coefficient, and the fins can be divided into straight fins, corrugated fins, etc. The fins not only increase the surface area of the heat exchange surface, but also promote fluid disturbance, enhancing heat exchange.

### Data source and performance evaluation

Based on the existing literature and our own research, the frosting amount of various freezing media is taken as a research subject as a whole, with more than 1800 sets of experimental data selected from 6 commonly used freezing media. Table 1 shows the source and distribution of experimental data. Of the experimental data used to train, verify, and test the dimensionless parameter-neural network model, there are 138 sets of R12, 670 sets of R134a, 249 sets of R22, 531 sets of R410A, and 43 sets of R407C, and 134 sets of R600a used for training and verification, and the remaining 140 sets are used for testing. MATLAB (R2019a) is used as a mathematical tool throughout the process.

RETRACTED

**Table 1:** Data sources and those for neural network training.

Freezing media	The amount of data	Training/testing
**R22**	47	Training 249
	110	Test 20
	112	-
**R12**	153	Training 138 Test 15
**R600a**	149	Training 134 Test 15
**R134a**	405	Training 670
	50	Test 50
**R410A**	215	-
	210	Training 531
	338	Test 40
**R407C**	23	-
	21	Training 43
	27	Test 5

The number of hidden layers varies from 3 to 15, and then, the traditional least square method used to compare the error is optimized. The optimized one can calculate the mean square error between all hidden layers in the same neural network, and then, the layer with the smallest mean square error is selected. The performance is evaluated, using mean square error (MSE), Root Error (RE), and root mean square error (RMSE).


$$MSE=1/(N-1)\sum_{i=1}^{N}\left[(X_{p}-X_{e})/X_{e}\right]$$ (11)

$$RE=1/N\sum_{i=1}^{N}(X_{p}-X_{e})/X_{e}$$ (12)

$$RMSE=\sqrt{1/(N-1)\sum_{i=1}^{N}{\left[(X_{p}-X_{e})/X_{e}-RE\right]}^{2}}$$ (13)

Where *X*_*p*_ and *X*_*p*_ represent the predicted value and experimental value, respectively; *N* represents the number of samples.

## Result analysis

### Model performance testing

To determine the optimal algorithm, Levenberg-Marquardt (LM) optimization algorithm [32], Bayesian regularization algorithm [33], and adaptive momentum gradient descent algorithm [34] are compared, as shown in Table 2. The adaptive learning rate (0–1) is incorporated in different algorithms to calculate the error, and the best learning rate is automatically selected. The minimum error is selected as the optimal algorithm for this training. It is noted from the table that, under the same number of optimal hidden layers, the adaptive momentum gradient algorithm has lower errors in RE, MSE, and RMSE, which are 0.0755, 0.0068, and 0.0827, respectively, and there are significant differences from other algorithms. There L-M optimization algorithm is basically consistent with the Bayesian regular optimization algorithm in RE, MSE, and RMSE. Finally, the adaptive momentum gradient algorithm is selected as the optimal network algorithm.

**Table 2:** Training results of different algorithms.

Different algorithms	Optimal hidden layer	Number of iterations	RE	MSE	RMSE
**L-M optimization algorithm**	6	35	0.1416	0.0388	0.1970
**Bayesian regularization algorithm**	6	174	0.1417	0.0414	0.2034
**Adaptive momentum gradient descent**	6	50	0.0755	0.0068	0.0827

As shown in Fig 5, in order to further determine the appropriate adaptive gradient algorithm, the AdaGrad (AD) [35], Momentum Stochastic (MS) [36], and Root Mean (RM) [37] algorithm are optimized. Fig 5A and 5B are the sensitivity analysis results of the hidden layer in the adaptive momentum gradient descent model. When the number of hidden layers is 6, the sensitivity analysis results of AD, MS and RM algorithms are 0.07, 0.00, and 0.08, respectively. Fig 5C and 5D are the weights and biases of the dimensionless parameters-neural network. It is noted that, the index weights of all layers are basically the same, and the overall structure of the model is optimal. Hence, when the number of hidden layers is 6, the overall sensitivity of the model is low, and the overall structure of the model is optimal.

RETRACTED

**Fig 5:** The sensitivity, weight, and bias of the hidden layer of the adaptive momentum gradient descent method. Fig A: the sensitivity, Fig B: the sensitivity coefficient, Fig C: the weight, Fig D: the bias, U-U6 are different neural network layers 1–6.

Fig 6A is the predicted value and experimental value after model training; Fig 6B is the predicted value and experimental value after model verification; Fig 6C is the relative error between the predicted value and the experimental value after model training; and Fig 6D is the relative error between predicted value and the experimental value after model verification. We further tested the actual prediction effects of the neural network and found that, after verification, the predicted value and experimental value showed obvious fluctuations. However, the fluctuation is significantly reduced after model training. It is calculated that, the mean square error of the dimensionless-neural network model is 1.68%, which is significantly reduced. Hence, the prediction performance of the optimized model has been significantly improved.

**Fig 6:** The training/verification performance and error results.

Fig 7A is a comparison between the predicted value of frost amount by the dimensionless parameter-neural network model and the experimental value using various refrigerants. It is noted that, the results of network training are generally satisfactory. The relative error between the predicted result and the actual output is within 7.55%, much better than 18.4% in the latest research. Therefore, the dimensionless parameter-neural network designed in this study is not only applicable to multiple refrigerants, but also has smaller errors. Fig 7B shows the prediction performance of the dimensionless parameter-neural network under different numbers of iterations, and the variation of the training value, the verification value, and the test value with the number of iterations. The target mean square error set before training is 10^−5,^ but the built-in verification error reaches its target error prematurely, and when the number of iterations reaches 42, the mean square error of the training model is 0.019827. Hence, the model constructed in this study is not only applicable to multiple refrigerants, but also has smaller errors.

RETRACTED

**Fig 7:** Model performance and errors under different freezing media.

As shown in Fig 8, the number of verifications is usually set to prevent overfitting of the training network. When the verification error is greater than the training error, the operation is stopped after the default verification number of 6 times is reached. As the number of iterations increases, the gradient of the model shows a trend of first rising and then falling, and after a brief fluctuation, the error basically stabilizes. The error remains basically stable under the first 40 iterations, and then it increases subsequently. It explains why that the training network stops running before it reaches the set mean square error of 10^−5^.

**Fig 8:** The training gradient size, error, and verification times. Fig A: the gradient size, Fig B: the error, Fig C: the number of verifications.

### Regression analysis

As shown in Fig 9, in order to further clarify the relationship between the predicted value of the model and the output value under different data sets, a regression analysis is conducted on the data of different data sets. Fig 9A–9D show the regression function between the network training, verification, and predicted output value. In each sub-figure, the dotted line represents the ideal correlation between the output value (predicted value) and target value (test value). The solid line represents the actual optimal linear correlation fit between the output value (predicted value) and target value (test value). The circle represents the target value of the actual output. The R value in the figure represents the correlation between the output value and the target value. A larger R value indicates that, the output value is closer to the target value. It is noted that, the output R values are 0.99993, 0.98792, and 0.99996 respectively, all close to 1, indicating that the fitted compressor neural network is reliable and highly accurate. In addition, it is found that, under different data sets, there is a strong correlation between the predicted value and the output value of the model, which further proves the effectiveness of the model proposed in this study.

**Fig 9:** Regression function between network training, verification and prediction output values. Fig A: the model result under the training data set, Fig B: the model result under the verification data set, Fig C: the model result under the test data set, and Fig D: the sum test result of all data.

RETRACTED

### Heat transfer characteristics simulation

As shown in Fig 10, the condenser outlet temperature of the original unit is higher than that of the new unit. The reason is that, the built-in electric auxiliary heating device of the original unit heats the air flowing out of the condenser outlet, while the condenser outlet of the new unit does not have an electric auxiliary heating device heating air. However, the difference in the outlet air temperature is not large. After calculations, during the entire process (120min), the original unit is only 0.72°C higher than the average temperature of the condenser outlet air of the new unit. The small difference in air temperature can shows the superiority of the new unit. In fact, out of consideration for the comfort, the defrosting methods of the two units can be combined to increase both COP and heat capacity. Under the conditions of dry bulb temperature/wet bulb temperature 2°C/98% (120min), compared with the original unit, the COP of the new unit increases by 21.86% in average, and the input power is lower by 25.63%, while the average heating capacity of the original unit (equipped with 2100W built-in electric-heating system) is only 8.25% higher than that of the new unit (including new defrost technology, front 320W, rear 160W, not using the built-in electric-heating system), and the average air temperature at the condensation outlet is also only 0.72°C higher than that of the new unit. This suggests that, when the built-in electric-heating equipment is removed, the heating capacity and outlet air temperature of the new unit are almost equal to those of the original unit, while the COP and the input power are significantly improved. In addition, the original unit experiences two frost-defrost processes during the entire test period, while the new unit only experiences once. Although the new unit delays frosting phenomenon but does not prevent it from occurring. It is fund that under this working condition, the amount of electric auxiliary heat of the front-mounted system is lower than the ideal minimum anti-defrosting energy, which indicates insufficient electric auxiliary heat. This also explains why the new unit still frosts once although the defrost problem has been greatly improved.

**Fig 10:** Heat transfer characteristics under working condition 1 at different times. Fig A: Coefficient of Performance (COP), Fig B: heating capacity, Fig C: input power, Fig D: condenser outlet air temperature.

As shown in Fig 11, the environmental conditions are set as follows: the dry bulb temperature is 6°C, and the wet bulb temperature is 68%. After actual testing, it is found that the original unit has higher heat capacity under this non-frosting condition. It is because the built-in electric auxiliary heating device (2100W) in the original unit endows the air flowing into the room with higher temperature and enthalpy value. After calculation, the average heat capacity of the original unit is only 6.57% higher than that of the new unit. During the entire test process (120min), the input power consumption of the original unit is 15.90% higher than that of the new unit. Similar to condition 1, the excessive input power of the original unit also explains why the newer unit has a higher heat capacity, but a smaller COP. Due to the high built-in electric auxiliary heating device of the original unit, the condenser outlet air temperature of the original unit is 3.22°C higher than that of the new unit during the entire test. It is noted from the figure that, the new unit has a higher COP under the two working conditions, and it is more energy-efficient and has smaller input power consumption. Although the original heat pump unit has higher heat capacity and condenser outlet air temperature, the results of the two groups are not much different, and in the long run, a small increase in heat capacity and a small increase in condenser outlet temperature at the cost of huge energy consumption id not cost-effective. In addition, under dry bulb temperature/wet bulb temperature 2°C/98%, the electric auxiliary heat of the front-mounted system is lower than the ideal minimum defrost energy, which indicates insufficient front-mounted electric auxiliary heat. This also explains why the new unit still frosts once despite the great improvement. In the following, the two methods can be combined so that the defrost heat pump increases the temperature of the indoor air and improves the thermal comfort.

RETRACTED

**Fig 11:** Heat transfer characteristics under working condition 2 at different times. Fig A: the training data set, Fig B: the verification data set, Fig C: the test data set, and Fig D: the sum test result of all data.

## Conclusions

Aimed at the frosting problem of the air source heat pump in low-temperature and high-humidity environment, the frosting characteristics at the evaporator side of the air source heat pump system are analyzed first; then, a new defrosting system is proposed, and its thermodynamics and heat transfer performance are simulated. Based on general frosting prediction correlation equations, the dimensionless parameter-neural network is proposed to predict the frosting amount. Its relative error is 7.55%, the mean square error is 0.68%, and the root mean square error is 8.27%. It is more flexible, more objective, and reliable in the selection of hidden layers, the acquisition of the optimal function, and the selection of the appropriate learning rate. The analysis of the performance of the new unit with anti-defrost device and the original unit with built-in electric auxiliary heating device reveals that, the COP of the new unit is 21.86% and 10.63% higher than that of the original unit under the two working conditions, and the input power is 25.63% and 15.90% lower than that of the original unit. When operating under low temperature conditions, the new unit has improved performance. However, some limitations should be noted in the study. For example, due to the interaction of the components, the freezing media, and the environment during the operation of the heat pump system, it is inevitable that the frosting amount on the heat exchanger will not be evenly distributed. Therefore, in the follow-up, a comparative study of the auxiliary heat is necessary, and a new heat pump evaluation method is needed according to thermal comfort needs. Additionally, the coupling between the anti-defrost control and the electric auxiliary heating device in the new unit with the original unit needs to be further explored.

## Supporting information

S1 Data (ZIP)
